# Effects of Ozone on Hippocampus BDNF and Fos Expressions in Rats with Chronic Compression of Dorsal Root Ganglia

This article has been retracted.

**DOI:** 10.1155/2021/5572915

**Published:** 2021-11-26

**Authors:** Lingling Zhu, Yanxiu Wang, Xiaowen Lin, Xu Zhao, Zhi jian Fu

**Affiliations:** ^1^Department of Pain Management, Provincial Hospital Affiliated to Shandong University, Shandong University, 324 Jingwu Road, Jinan, Shandong 250021, China; ^2^Department of Pain Management, Taian City Central Hospital, 29 Longtan Road, Taian, Shandong 271001, China

## Abstract

The effects of ozone on hippocampal expression levels of brain-derived neurotrophic factor (BDNF) and c-fos protein (Fos) were evaluated in rats with chronic compression of dorsal root ganglia (CCD). Forty-eight adult female Sprague-Dawley rats were randomly divided into the following 4 groups (*n* = 12): sham operation (sham group), CCD group, CCD with 20 *μ*g/ml of ozone (CCD + AO_3_ group), and CCD with 40 *μ*g/ml of ozone (CCD + BO_3_ group). Except the sham group, unilateral L5 dorsal root ganglion (DRG) compression was performed on all other groups. On days 1, 2, and 4 after the operation, the CCD + AO_3_ and CCD + BO_3_ groups were injected with 100 *μ*l of ozone with concentrations of 20 and 40 *μ*g/ml, respectively. Thermal withdrawal latencies (TWLs) and mechanical withdrawal thresholds (MWTs) were measured at various time points before and after the operation. BDNF and Fos expressions were examined in the extracted hippocampi using immunohistochemistry. The TWLs and MWTs of CCD model rats that received ozone were lower with decreased BDNF and increased Fos expression levels, on day 21 after the operation, compared to those of the sham group (*P* < 0.05). The TWLs and MWTs of the CCD + AO_3_ and CCD + BO_3_ groups were higher with increased BDNF and decreased Fos expression levels, on day 21 after the operation, compared to those of the CCD group (*P* < 0.05). The TWLs were longer and the MWTs were higher in the CCD + BO_3_ group at each time point with increased BDNF and decreased Fos expression levels, on day 21 after the operation, compared to those of the CCD + AO_3_ group (*P* < 0.05). Our results revealed that ozone can relieve the neuropathic pain caused by the pathological neuralgia resulting from DRG compression in rats. The mechanism of action for ozone is likely associated with changes in BDNF and Fos expression levels in the hippocampus.

## 1. Introduction

Since its first use in 1988, ozone has been widely used to treat pain in many diseases. Lumbar and leg pain have been treated with epidural ozone injection in clinical studies; however, its specific mechanism is still unclear. As a classical model of neuropathic pain, chronic compression of dorsal root ganglia (CCD) simulates the lumbar and leg pain caused by clinical disc herniation and intervertebral foramen stenosis [1]. Previous studies have shown that the hippocampus is a crucial area affected by pain stimulation and involved in pain signal processing [2, 3].

Rat hippocampi usually comprise two regions, CA1 and CA3. The CA1 region is an especially sensitive region; cerebral ischemia has been reported to selectively damage hippocampal CA1 neurons, while keeping neurons in other subfields undamaged [4, 5]. The CA1 region has been shown to be closely associated with the occurrence and development of chronic pain. For instance, formalin-induced inflammatory pain stimulation has been shown to increase the probability and amplitude of long-term potentiation (LTP) induction in the DG and CA1 regions, which could be completely abolished by blocking nociceptive inputs at the peripheral injury site [6]. Microinjecting N-methyl-D-aspartic acid receptors (NMDARs) inhibitors into the CA1 region has been shown to significantly inhibit chronic pain.

Brain-derived neurotrophic factor brain-derived neurotrophic factor (BDNF) and c-fos protein (Fos) are expressed abundantly in the hippocampus. BDNF is a polypeptide secreted by nerve cells and target tissues. Fos is a well-established marker of pain pathway activation. Under painful stimuli, a decreased BDNF level induces the autophosphorylation of tyrosine protein kinases, thereby activating ERK1/2 through a series of cascades into p-ERK1/2 and transporting it from the cytoplasm into the nucleus. The aforementioned processes promote the transcription and expression of certain genes including c-fos, which initiates cell proliferation and differentiation while playing an important role in cell growth, development, and proliferation. Acute or chronic pain has been shown to significantly reduce the levels of *BDNF* mRNA [7]. t-5224, an inhibitor of c-fos, has been found to alleviate spared nerve injury- (SNI-) induced pain responses in mice. Studies have also shown that spinal c-fos expression can be reduced by analgesic drug application [8, 9].

This study evaluated the effects of epidural ozone injection on pain threshold and hippocampus expressions of BDNF and Fos in a CCD rat model to elucidate the mechanism of ozone therapy in lumbar and leg neuralgia, thereby providing an experimental basis for clinical application.

## 2. Materials and Methods

### 2.1. Animal Selection and Grouping

In total, 48 healthy female 8-week-old rats weighing 250~280 g were procured from Beijing Huafukang Biotechnology Co., Ltd. and acclimatized at 20–25°C for 24 hours. These rats were randomly divided using digital tables into the 4 following groups (*n* = 12): sham group, CCD group, CCD model with 20 *μ*g/ml ozone (CCD + AO_3_) group, and CCD model with 40 *μ*g/ml ozone (CCD + BO_3_) group.

### 2.2. Model Preparation and Epidural Catheterization

Apart from the sham group, the CCD model was induced in all other groups, as described by Song et al. [1]. Rats were anesthetized by intraperitoneally injecting sodium pentobarbital. Then, the lumbosacral region was routinely shaved and disinfected before a posterior median left lateral incision was made along the rat spinous process, and the skin was incised from the left border of the L4-L6 vertebrae, followed by blunt separation to the transverse process. Once the extraforaminal foramen at the root of the transverse process is exposed, cephalad insertion of a needle (bent at 90°) into the foramen was performed at angles of 30°and 10° to the median and the spinal horizontal lines, respectively. The needle was withdrawn once the nerve root palpation caused a slight tic in the ipsilateral hindlimb muscles. Subsequently, a stainless-steel column with a length of 6 mm and a diameter of 0.6 mm was inserted into the intervertebral foramen along the needle to ensure constant compression of the adjacent nerve roots. The muscles and low back fascia were then sutured sequentially. For rats in the sham group, no steel column compression was applied after identifying the intervertebral foramen position. The method described by Nishiyama [10] was used to place the outer tube of the hard film for each group. After determining the position of the T13/L1 gap and separating the interspinous and ligamentum flavum from the intervertebral space, a 13 cm long PE catheter was inserted at one end 1.5 cm caudally and secured to the adjacent muscles using silk sutures. The neck skin was incised by 0.5 cm to create a subcutaneous tunnel; the PE catheter was secured to the neck with a transcutaneous tunnelled silk suture at the other end. After the operation, normal saline was used to flush the incision, before the back fascia and skin were sutured. Rats in each group received penicillin intraperitoneally to prevent infection. After remaining awake for 2 hours, rats from all groups were returned to single cage housing in the animal holding room. On days 1, 2, and 4 after surgery, the rats in the CCD + AO_3_ and CCD + BO_3_ groups were injected with 100 *μ*l each of ozone through the epidural catheter at concentrations of 20 and 40 *μ*g/ml, respectively.

### 2.3. General Behavioural Observation

Health statuses and activity levels of rats were continuously observed. Changes in skin, muscle tone, posture, and gait of the hind limbs on the operated side of rats were recorded daily. Rats with no ulceration, paralysis, and autophagic limbs were selected for subsequent tests.

### 2.4. Determining Thermal Withdrawal Latency (TWL)

TWL was detected on the day before the operation as well as 1, 3, 5, 7, 14, and 21 days after the operation. According to the method described the Hargreaves [11], a BME-410C type thermal pain stimulator was used for testing, which was developed by Institute of Biomedical Engineering, Chinese Academy of Medical Sciences. Rats were placed over a 3 mm thick plexiglass plate with the thermal pain stimulator placed below. The light source was focused to illuminate the plantar skin corresponding to the 4^th^ and 5^th^ metatarsals on the postoperative rat hind limbs. The latency from the initiation of illumination up until the appearance of hindlimb withdrawal responses was determined as the sensitive observation indicator of heat-induced pain. Measurements were repeated 3 times at 5 min intervals; the mean for each rat was used for statistical analysis.

### 2.5. Detection of Mechanical Withdrawal Threshold (MWT)

The mechanical withdrawal threshold (MWT) was measured on the day before the surgery as well as 1, 3, 5, 7, 14, and 21 days after the surgery. Four hours after the TW measurements, the mechanical pain threshold was measured using von Frey filaments (up-down method) [12]. Rats were placed inside a clear Plexiglas box for detection; the skin corresponding to the 4^th^ and 5^th^ metatarsal bones of the rat left hind foot was perpendicularly stimulated with von Frey cilia with different folding forces (in ascending order). The cilia were bent into a sigmoid shape and maintained for 6 ~ 8 s at 30 s intervals. Positive responses of the rats included rapid withdrawal of hind foot, flinching, and other phenomena. If a positive response was not observed in a rat after stimulation, then, ciliary restimulation with a higher force is applied. Ciliary stimulation was repeated 5 times for each force. The minimum intensity that elicited more than three positive responses was recorded. If no positive response was observed in rats upon application of the maximum cilial force, then, this maximum force was used for subsequent calculations. The following specific formula was used to calculate MWT: (10^[*xf* + *κδ*]^)/10000 where *xf* is the logarithmic value of the last used force; *κ* is the coefficient under different stimulation conditions, and *δ* has a fixed value of 0.224.

### 2.6. Nissl Staining

Six rats were randomly selected from the CCD and CCD + BO_3_ groups and abdominally anesthetized using 10% hydrochloraldehyde (0.38 mL/100 g). The heart was perfused with 50 ml of 4% paraformaldehyde/0.1 mol/L phosphate buffer, and the dorsal root ganglion (DRG) of L5 was removed and fixed with 4% paraformaldehyde for 24 h. After routine dehydration and paraffin embedding, serial sections were taken. Sections approximately 4 *μ*m thick were extracted until the entire hippocampus was removed. Sections were stained with cresyl violet (Nissl staining) for 50 s, dehydrated, diaphanized, and mounted for observation. Cell counting was performed in three adjacent DRG sections. Only cells with visible nuclei and nucleoli were counted. Five visual fields were randomly selected, and images were captured from each slice in the cerebral cortex area (400 power microscope). The number of living cells in each high-power microscope visual field was determined.

### 2.7. Immunohistochemical Examinations

The process of obtaining sections is the same as Nissl staining. Antibodies against BDNF (batch number: sc20981, Santa Cruz company, USA) and Fos (batch number: sc-271243, Santa Cruz company, USA) were diluted at 1 : 150. The cells were incubated overnight at 4°C in 50 *μ*l of the diluted antibody solutions. Cells were then incubated with the horseradish peroxidase-labelled secondary antibody for 30 min. PBS was used as the negative control instead of using primary antibody. Three sections were labelled by each antibody, and two nonoverlapping visual fields were randomly selected from each section in the target area. The average optical densities of BDNF and Fos in hippocampal tissues were measured using Image Pro Plus 6.0.

### 2.8. Western Blot Test

After the last pain threshold test, the rats were anesthetized with sodium pentobarbital. Six rats in each group were randomly selected and sacrificed with an intraperitoneal injection of 10% chloral hydrate (0.38 ml/100 g body weight). The hippocampal tissue on the operation side was extracted and stored in liquid nitrogen. Tissue samples were weighed, cleaned, and centrifuged. The ratio of protease inhibitor to the protein extraction reagent (precooling to 4°C) was 1 : 99. After 1 *μ*g of tissue was added to 10 *μ*l of tissue cell lysis solution, the tissue was homogenized, incubated on ice for 30 min, and then centrifuged at 12,000 rpm for 30 min at 4°C. The supernatant was collected, and the protein concentration was determined using the BCA method. The remaining protein supernatant was proportionally added to the loading buffer, mixed evenly, and denatured in 100°C metal bath for 10 min. Subsequently, it was cooled to room temperature and stored at −80°C. In total, 40 *μ*g of the protein samples was separated by 10% SDS-PAGE and transferred to PVDF membrane by wet electro-spinning. After sealing the membrane in 5% skimmed milk powder for 1 h at room temperature, the membrane was washed three times with TBST (tris buffered saline tween) for 5 min each. BDNF (1 : 1 000), Fos (1 : 500), and *β*-actin (1 : 1000) antibodies were was incubated with the membrane overnight at 4°C. The next day, the membrane was washed three times with TBST for 10 minutes each. The membrane was incubated with horseradish peroxidase-labelled secondary antibody (1 : 5000) at room temperature for 1 h. Subsequently, the membrane was washed 3 times with TBST for 15 min each. The ECL chemiluminescence method was used to image the protein bands. Image-Pro Plus 6.0 was used to quantitatively analyse the protein bands.

### 2.9. Statistical Analysis

The data were processed using the SPSS 22.0 statistical software, and the measured data were expressed as mean ± standard deviation. Values between two groups were compared using independent *t*-tests. One-way ANOVA was also used to compare between groups, and the Student Newman Keuls test was used to compare the sample means. *P* < 0.05 was considered statistically significant.

## 3. Results

### 3.1. Successful Establishment of the CCD SD Rat Model

Eight SD rats were preexperimental before formal experimentation, two died within 24 h and one within 72 h after surgery, so the mortality rate of rats was 0.75%. No further rat death occurred until the end of the formal experiment. After the formal experiment, we found that all CCD rats walked normally with no obvious gait alterations; no self-injurious behaviours were observed. All rats developed a frequent lifting action of the postoperative hind foot and licking. Therefore, the CCD model success rate was 100% in formal trials.

### 3.2. Epidural Ozone Injection Increases TWL

Compared to the preoperative values, there was no significant change in the TWL at each time point for the sham group (*P* > 0.05). On day 1, compared with those of the sham group, TWL values of the remaining groups decreased significantly (*P* < 0.05); however, there was no significant difference between the CCD model group and the groups that received ozone. Until the 5^th^ postsurgery day, the TWLs of CCD + AO_3_ group were not significantly different from those of the CCD group; however, the TWLs of CCD + BO_3_ group (day 3, mean ± SD = 6.96 ± 1.91; day 5, mean ± SD = 8.78 ± 2.43) were higher than those of the CCD group (day 3, mean ± SD = 4.91 ± 1.16, *P* = 0.005; day 5, mean ± SD = 5.71 ± 1.58, *P* = 0.002) and higher than those of CCD + AO_3_ group as well (day 3, mean ± SD = 5.37 ± 0.98, *P* = 0.013; day 5, mean ± SD = 6.18 ± 2.11, *P* = 0.004). This result suggested that a high concentration of ozone can significantly increase the thermal threshold from day 3 to day 5 after the operation. On the 7th day, TWL values of the CCD + AO_3_ (8.67 ± 0.99, *P* = 0.012) and CCD + BO_3_ groups (10.97 ± 2.47, *P* < 0.001) continued to increase and were significantly higher than that of the CCD group (6.35 ± 1.89, *P* < 0.001). After 14 and 21 days, the ozone intervention groups had significantly higher TWLs than that of the CCD group; TWLs for the CCD + BO_3_ group was also higher than those of the CCD + AO_3_ group (*P* < 0.05). These results showed the ozone significantly reduced the thermal pain threshold of rats with time. The effect of high concentration ozone on pain relief was higher than that of low concentration ozone. (Figure 1(a)).

### 3.3. Epidural Ozone Injection Increases MWT

Before surgery, there was no significant difference in MTW among all groups (*P* > 0.05). On days 1 and 3 days after the operation, the MWT values of other groups decreased significantly compared to that of the sham group (*P* < 0.05); however, there were no significant differences between model and intervention groups. On day 5 after operation, MWT of the CCD group (5.01 ± 0.98) had no significant change; however, the MWTs of the ozone intervention groups (CCD + AO_3_, 6.30 ± 1.53, *P* = 0.046; CCD + BO_3_, 6.80 ± 1.66, *P* < 0.018) were higher than that of CCD group. There were no significant differences between the CCD + AO_3_ and CCD + BO_3_ groups. On the 7^th^ day after the operation, the MWT value of the ozone intervention groups (CCD + AO_3_, 7.19 ± 1.29, *P* < 0.001; CCD + BO_3_, 8.78 ± 1.31, *P* < 0.001) continued to increase, which was significantly higher than that of the CCD group (5.11 ± 1.25). The CCD + BO_3_ group had a higher MWT than that of the CCD + AO_3_ group on day 7 postsurgery (*P* < 0.01). On days 14 and 21 after the operation, the MWTs for the ozone intervention groups were significantly higher than those of the CCD group; the MWT of the CCD + BO_3_ group was higher than that of the CCD + AO_3_ group (*P* < 0.01). These results showed that ozone group significantly reduced the mechanical pain threshold of rats with time. Moreover, the effect of high ozone concentration was higher than that of low ozone concentration (Figure 1(b)).

### 3.4. Ozone Improves the Morphology and Number of DRG Cells after CCD

Under normal conditions, the DRG cells are morphologically regular and closely arranged. Nissl bodies of DRG neurons are dark blue dense granules. In the CCD group, DRG cells were shrunken with indistinct cytoplasm, loose arrangement, and faint staining (Figure 2(a)). After ozone intervention, not only did the number of DRG cells increase, but the Nissl staining also became darker compared to that in the CCD group (Figure 2(b)). Sensitive neuronal survival was investigated by counting the number of L5 DRG neurons. Ozone treatment also led to an obvious reduction in neuronal preservation. The number of DRG neurons in the CCD + BO_3_ group (73.5 ± 16.5) was significantly higher than that in the CCD group (42.6 ± 12.33) (*P* < 0.01) (Figure 2(c)). This result indicated that ozone improves the morphology and number of dorsal root ganglion cells after CCD.

### 3.5. Immunohistochemical Results

#### 3.5.1. Average Optical Density of BDNF Significantly Increases in Hippocampal Cells after Epidural Ozone Injection

Visual naked-eye observation of the brown staining revealed that BDNF is mainly expressed in the cytoplasm and on the cell membrane of hippocampal cells in each group. Although it was lower than that of the sham group (Figure 3(a)), the staining intensity was higher in the CCD + BO_3_ group (Figure 3(d)) than in the CCD + AO_3_ group (Figure 3(c)), which in turn was higher than that in the CCD group (light stain) (Figure 3(b)). The average optical density of BDNF in the CCD group (0.14 ± 0.038) was lower than that in the sham group (0.37 ± 0.045) (*P* < 0.001), whereas those in the CCD + AO_3_ (0.21 ± 0.043) and CCD + BO_3_ groups (0.28 ± 0.049) were higher than that in the CCD group (*P* < 0.05). The expression level of BDNF in the CCD + BO_3_ group was notably higher than that in CCD + AO_3_ group (*P* = 0.012); however, it was still lower than that in the sham group (*P* = 0.002) (Figure 3(e)).

#### 3.5.2. Average Optical Density of Fos Significantly Decreases in Hippocampal Cells after Epidural Ozone Injection

Brown staining representing Fos was mainly concentrated in the nuclei. Although it was higher than that in the Sham group (Figure 4(a)), the degree of staining in the CCD + BO_3_ group (Figure 4(d)) was lower than that in the CCD + AO_3_ group (Figure 4(c)), which in turn was clearly lower than that in the CCD group (Figure 4(b)). The average optical density of Fos in CCD group (0.40 ± 0.065) was higher than that in the sham group (0.13 ± 0.048) (*P* < 0.001). The average optical densities of Fos in the CCD + AO_3_ (0.29 ± 0.058) and CCD + BO_3_ groups were lower than that in the CCD group (*P* < 0.05). The average optical density in the CCD + BO_3_ group was also lower than that in CCD + AO_3_ group (*P* = 0.043); however, it was still higher than that in the sham group (*P* = 0.003) (Figure 4(e)).

### 3.6. Gray Values of BDNF and Fos Are Significantly Elevated in Hippocampal Cells after Ozone Intervention

Analysis of the BDNF gray values revealed that although the BDNF level in the CCD + BO_3_ group (0.76 ± 0.18) was lower than that in the sham group (1.01 ± 0.25) (*P* = 0.021), it was higher than that in the CCD + AO_3_ group (0.52 ± 0.14) (*P* = 0.026), which in turn was higher than that in the CCD group (0.29 ± 0.07) (*P* < 0.001). Analysis of Fos gray values revealed that the expression of CCD group (1.19 ± 0.23) was higher than that of the sham group (0.42 ± 0.11) (*P* < 0.001), with downregulated levels in the CCD + AO_3_ (0.96 ± 0.10) and CCD + BO_3_ group (0.70 ± 0.19) (*P* < 0.05). The expression of Fos in the CCD + BO_3_ group was significantly lower than that in the CCD + AO_3_ group (*P* = 0.014); however, it was still higher than that in the sham group (*P* = 0.009) (Figure 5).

## 4. Discussion

As the recognition of the effectiveness of medical ozone therapy in pain management increases, its detailed mechanism is also being investigated. The DRG is the aggregation site for primary sensory afferent neurons. Abnormal electrical activity after an injury triggers persistent neuropathic pain and is crucially involved in pain signal transduction [13]. Although clinical research has shown that the administration of ozone effectively alleviates neuropathic pain caused by damage to the DRG, its related mechanism has not yet been elucidated. Long-term chronic injury to the DRG has been reported to be involved in central sensitization closely related to hyperalgesia and allodynia [14, 15]. The hippocampus, which is the limbic system of the brain, is an important structure involved in the relevant integrative processing of this pain information. Therefore, this study assessed the damage to the DRG and the alteration of crucial hippocampal protein levels after ozone intervention to elucidate the mechanism by which ozone reduces pain.

In this study, once the CCD model was established, the rats exhibited pain-induced abnormalities such as toe apposition, lifting, and licking. The threshold between the thermal and mechanical paw withdrawal responses of rats in the CCD group was significantly lower than that in the sham group at all observed time points after the surgery, suggesting the occurrence of thermal and mechanical pain sensitivity, thereby indicating the successful establishment of the model. Numerous studies have shown that although ozone exhibits antioxidation and anti-inflammatory effects to treat diseases, it can also aggravate oxidative stress or lead to disease [16]. In this preliminary study found that 20 *μ*g/ml of O_3_ did not affect the survival of spinal cord cells, whereas ozone concentrations of 30 to 100 *μ*g/ml have been shown to be concentration-dependently neurotoxic to spinal cord neurons [17]. Intrathecal injection of ozone at concentrations of 10, 20, or 30 *μ*g/mL has been shown to significantly reduce mechanical PWT; ozone concentration of 20 *μ*g/ml could not induce nerve damage and was reported to have an anti-inflammatory effect [18]. Ozone at high concentrations of 40, 60, and 80 *μ*g/ml can cause neural apoptosis and peroxide damage through the JNK/MAPK signalling pathway, causing significant neurotoxicity. Therefore, this study selected epidural ozone injection that increased the arachnoid barrier. The effects of ozone at concentrations of 20 and 40 *μ*g/ml on the operative toe pain threshold were assessed after damaging the DRG.

The results of this study suggested that the thermal paw withdrawal response period of the operated rat foot was significantly longer, and the threshold of mechanical paw withdrawal response was significantly improved after ozone intervention compared to those of the CCD group, suggesting that ozone intervention alleviated thermal and mechanical pain sensitivity in rats. Our results also suggested that ozone at a concentration of 40 *μ*g/ml increased the pain threshold more significantly than that at 20 *μ*g/ml. We believe that 40 *μ*g/ml ozone has a protective effect rather than a toxic effect because of the arachnoid as a barrier.

Expression of Fos is the central response to various noxious stimuli, and its expression levels are positively correlated with the intensity of the stimulation [19]. As a marker of nociceptive pain conduction, Fos can be widely used to explore pain conduction pathways and investigate pain modulation [20, 21]. In this study, the protein expression levels of Fos in the CCD model group were significantly higher than those in the control and ozone intervention groups. Fos expression in the CCD model was downregulated by ozone intervention. The degree of downregulation by ozone concentration of 40 *μ*g/ml was more pronounced than that by 20 *μ*g/ml, which was consistent with the changes in thermal and mechanical hyperalgesia in each group. These results suggested that the pain induced by CCD can alter the levels of pain-related factors in the hippocampus.

Levels of BDNF, which are abundant in the hippocampus, also change significantly by the process of chronic pain. BDNF has been shown as a critical mediator of central sensitization and an important regulator of neuronal excitability and plasticity [22–24]. BDNF is also involved in different pain models such as inflammation-induced hyperalgesia [25], complete Freund's adjuvant-induced thermal hyperalgesia [26], mechanical hyperalgesia in an L5 anterior rhizotomy model [27], and a spinal nerve ligation model [28]. Currently, chronic pain in peripheral tissues is believed to be equivalent to persistent stressors, which can cause apoptosis of neurons and decrease hippocampal BDNF expression; this indicates that peripheral noxious stimulation can regulate BDNF expression in the higher brain centre [29, 30]. Our results revealed that the BDNF protein expression in the CCD model group was significantly lower than that in the control group. Ozone concentration of 40 *μ*g/ml induced a more pronounced upregulation than that by 20 *μ*g/ml. This result indicated that ozone probably increased the pain threshold by upregulating hippocampal BDNF expression. However, BDNF expression levels in the DRG, spinal cord, and brain centre are different. In an SNI model, the BDNF levels in the DRG neurons of damaged nerves are upregulated, whereas that of undamaged nerves is downregulated [31]. CFA has been shown to increase BDNF expression and phosphorylated ERK in the spinal dorsal horn; the ERK inhibitor, U0126, has also been reported to reverse the increase in pain sensitivity [32]. In a chronic constriction injury (CCI) state, BDNF and MAPK expression levels in the spinal dorsal horn have been shown to increase, which could be inhibited by a MAPK inhibitor, thereby hindering pain sensitization [33, 34]. Ma et al. [35] have shown that elevating BDNF expression levels has been shown to reverse electrophysiological disturbances in vCA1-IL connectivity, alleviating spontaneous pain, thereby promoting a full recovery from pain.

Studies have found that there is some correlation between BDNF and Fos. c-fos, which forms a heterodimer with c-Jun, acts on the AP-1 site of target genes to regulate target gene expression, while BDNF contains an AP-1 site in its gene regulatory sequence, which may be regulated by Fos [36, 37]. Kim et al. [38] found that the addition of BDNF to spinal neuron culture fluid caused a rapid increase in c-fos mRNA. Spinal c-fos expression was also markedly increased 3 h after intrathecal BDNF injection in adult rats [39]. However, another study found that deletion of c-fos did not affect the expression of BDNF mRNA in CA1 and CA2 regions compared with c-fos mutated mice and wild type [40]. Thus, the interrelationship of BDNF and Fos expression is not clear. In this experiment, whether there is a correlation between the increase of BDNF expression and the decrease of Fos under the intervention of ozone remains to be further studied.

In conclusion, Epidural ozone could reduce chronic pain caused by long-term damage to the dorsal root ganglia, which is likely associated with hippocampal BDNF and Fos expression. Future studies will explore the signal pathway through which ozone interferes with the expression of BDNF and Fos.

## Figures and Tables

**Figure 1:** Effect of epidural ozone injection in alleviating pain in CCD model SD rats. With CCD, the thermal withdrawal latency (TWL) and mechanical withdrawal threshold (MWT) significantly reduced from day 1 to day 21 postsurgery (*P* < 0.001 for both) ((a) and (b)). The thermosensitive pain was alleviated between day 7 and day 21 after surgery in the CCD + AO_3_ group (*P* < 0.05 for all except day 10, where *P* = 0.002). The thermosensitive pain was significantly alleviated in the CCD + BO_3_ group between day 3 and day 21 after surgery (*P* < 0.001 for both). The thermosensitive pain-relieving effect between day 3 and day 21 postsurgery was more pronounced in the CCD + BO_3_ group than in the CCD + AO_3_ group (*P* < 0.001 for both) (a). The mechanical allodynia was alleviated between day 7 and day 21 in the CCD + AO_3_ group (*P* < 0.01 for all except day 7, where *P* = 0.046). The mechanical allodynia was also relieved significantly in the CCD + BO_3_ group between day 5 and day 21 (*P* < 0.001 for all except day 5, where *P* = 0.018). The thermosensitive pain-relieving between day 7 to day 21 was more pronounced in the CCD + BO_3_ group than in the CCD + AO_3_ group (*P* < 0.001) (b). Data are expressed as mean ± SD (^a^*P* < 0.05 and ^aa^*P* < 0.01, vs. sham group; ^b^*P* < 0.05 and ^bb^*P* < 0.01, vs. CCD group; ^c^*P* < 0.05 and ^cc^*P* < 0.01, vs. CCD + AO_3_ group).

**Figure 2:** In the CCD group, DRG cells were shrunken with indistinct cytoplasm, loose arrangement, and faint staining (Figure 2(a)). After ozone intervention, the number of DRG cells increased, while the Nissl staining became darker compared to those of the CCD group (Figure 2(b)). The number of DRG neurons in the CCD + BO_3_ group was significantly higher than that in the CCD group (*P* < 0.01) (Figure 2(c)).

**Figure 3:** BDNF was mainly expressed in the cytoplasm and on the membrane of hippocampal cells in each group, as represented by brown staining. The average optical density of BDNF in the CCD group was lower than that in the sham group (*P* < 0.001), whereas those in the ozone intervention groups were higher than that in the CCD group (CCD + AO_3_, *P* < 0.05; CCD + BO_3_, *P* < 0.01). The average optical density of BDNF in the CCD + BO_3_ group was higher than that in the CCD + AO_3_ group (*P* < 0.05); however, it was still lower than that of the sham group (*P* < 0.05). Data are expressed as mean ± SD (^a^*P* < 0.05 and ^aa^*P* < 0.01, vs. sham group; ^b^*P* < 0.05 and ^bb^*P* < 0.01, vs. CCD group; ^c^*P* < 0.05 and ^cc^*P* < 0.01, vs. CCD + AO_3_ group).

**Figure 4:** Fos staining, shown in brown, was mainly concentrated in the nucleus. Although it was lower than that in the CCD group (*P* < 0.01), the average optical density of Fos in hippocampal cells in the CCD + AO_3_ group was higher than that in the CCD + BO_3_ group (*P* < 0.05), which in turn was higher than that in the sham group (*P* < 0.01). Data are expressed as mean ± SD (^aa^*P* < 0.01 compared with the sham group; ^b^*P* < 0.05 and ^bb^*P* < 0.01, compared with the CCD group; ^c^*P* < 0.05 and ^cc^*P* < 0.01, compared with the CCD + AO_3_ group).

**Figure 5:** Western blot band images and quantitative determination of relative densities revealed that CCD of DRG significantly decreased the expression of BDNF in hippocampi compared to that in the sham group (*n* = 6/group). Epidural injection of ozone (20 or 40 *μ*g/ml) increased the protein expression of BDNF compared with that in the sham group (*n* = 6/group) (*P* < 0.05). Quantitatively, BDNF relative densities were calculated as the ratio of BDNF protein band intensity to that of actin. Ozone reduced the hippocampal expression of Fos. Western blot images and quantitatively calculated relative densities revealed that CCD of DRG significantly increased the hippocampal expression of Fos compared with that in the sham group (*n* = 6/group). Epidural injection of ozone (20 or 40 *μ*g/ml) decreased the protein expression of Fos compared to that in the CCD group (*n* = 6/group) (*P* < 0.05). Quantitatively, relative densities of Fos were calculated as the ratios of Fos protein band intensities to those of actin. Data are presented as mean ± SD (^aa^*P* < 0.01 vs. sham group; ^b^*P* < 0.05 and ^bb^*P* < 0.01, vs. CCD group; ^c^*P* < 0.05 and ^cc^*P* < 0.01, vs. CCD + AO_3_ group).

## Data Availability

The data used to support the findings of this study are available from the corresponding author upon request.
